# *Sonchus oleraceus* L. Promotes Gastroprotection in Rodents via Antioxidant, Anti-Inflammatory, and Antisecretory Activities

**DOI:** 10.1155/2022/7413231

**Published:** 2022-08-23

**Authors:** Cristian A. D. Vecchia, Gelvani Locateli, Patricia Z. Serpa, Denise Bianchin Gomes, Jackeline Ernetti, Daniela Miorando, Maria Eduarda D. C. Zanatta, Ruan Kaio Silva Nunes, Silvana M. Wildner, Max V. Gutiérrez, Wagner Vilegas, Lincon B. Somensi, Luisa M. Silva, Walter A. Roman Junior

**Affiliations:** ^1^Postgraduate Program in Health Sciences, Community University of Chapeco Region, 89809-900 Chapecó, SC, Brazil; ^2^Pharmacognosy Laboratory, Community University of Chapecó Region, 89809-900 Chapecó, SC, Brazil; ^3^Postgraduate Program in Pharmaceutical Sciences, University of Vale do Itajaí, Itajaí, SC, Brazil; ^4^Institute of Biosciences, São Paulo State University, Campus Litoral Paulista, 01049-010 São Vicente, SP, Brazil; ^5^Postgraduate Program in Development and Society, Alto Vale do Rio do Peixe University, 89500-000 Caçador, SC, Brazil

## Abstract

*Sonchus oleraceus* L. is an edible and medicinal plant used to treat stomachache and gastric ailments around the world. Thus, this study aimed to determine the gastroprotective mode of action of hydroalcoholic extract of *S*. *oleraceus* (HES). Mice were treated with HES before induction of gastric ulceration by ethanol/HCl. The area and histological appearance of ulcers were quantified, and mucus was measured histochemically. The effects of HES on inflammatory and oxidative markers were assessed in the ulcerated tissue. In addition, we investigated the gastric acid antisecretory activity of HES in pylorus-ligated rats. Chemical analyses of HES and its antioxidant activity were also performed *in vitro*. The HES (30 or 300 mg/kg) reduced the ulceration by 71.5 and 76.2%, respectively, compared with vehicle (*p* < 0.001), and the histological analysis confirmed the macroscopic results with elevation in mucin levels by 361.4 and 477.5%, respectively, compared with vehicle (*p* < 0.001). Moreover, the gastroprotection was accompanied by increases in GSH levels and in SOD, CAT, and GST activities; in parallel to a reduction in MPO activity and TNF levels. Furthermore, HES reduced the total acidity, and pepsin activity of the gastric juice of rats by 61 and 63%, respectively, compared to the vehicle. Phytochemical analysis indicated that luteolin-7-*O*-*β*-D-glucoside is the main active compound annotated in HES. Was also found that HES scavenged the DPPH radical with an IC_50_ of 15.41 *μ*g/mL. In conclusion, the gastroprotective effects of HES involve reductions in oxidative stress and inflammatory injury, in conjunction with an increase in mucus layer and inhibition of gastric secretion. This study advances in elucidating the modes of the antiulcer potential of *S*. *oleraceus* and contributes to the prospection of new gastroprotective molecules.

## 1. Introduction

Gastric ulceration is a mucosal-type injury that can involve the entire thickness of the gastric mucosa and thereby extend to the underlying muscle layer [1, 2]. This disease is a prominent global health problem associated with a multifactorial etiology and a complex repair process [3]. The development of such gastric lesions can be attributed to an imbalance in gastric homeostasis between aggressive agents, such as acid secretion, reactive oxygen species (ROS), and pepsin, and protective factors, including the mucus barrier, bicarbonate secretion, antioxidant defenses, and adequate blood flow [4].

In response to marked increases in aggressive agents associated with certain triggering factors, including social stress, alcoholism, smoking, a poor diet, *Helicobacter pylori* infection, prolonged use of non-steroidal anti-inflammatory drugs, and the inefficient operation of appropriate defense mechanisms, ulcerous lesions can occur in the epithelial wall of the gastric mucosa [5]. In this regard, ethanol consumption has been established to promote reductions in the integrity of mucus production, cell proliferation, and mucosal blood circulation, which in turn causes an escalation in ROS production and thereby induces an intense inflammatory response [6, 7]. Consequently, acidified or non-acidified ethanol has routinely been employed as an ulcerogenic agent in experimental studies to evaluate the gastroprotective activity of substances.

The treatment of gastric ulcers is based on a reduction of acidity in the gastric luminal content, involving proton pump inhibitors (e.g., omeprazole), and histamine *H*2 receptor antagonists (e.g., ranitidine) [3, 8], or antacids [9]. Furthermore, gastric ulcers associated with *H*. *pylori* infection require treatment based on the administration of antibiotics. However, despite the efficacy of such agents, their use is often associated with certain adverse side effects [10–12]. Moreover, given the high incidence of ulcer recurrence and the development of tolerance or preneoplasia injury in the gastric mucosa [13], there has been an intensification of studies that seek to identify safe and effective alternative resources, with a particular focus on the antiulcerative potential of natural products [14].

The leaves of *Sonchus oleraceus* L. (Asteraceae), a species native to Europe that now has a global distribution, are widely consumed in some regions of Asia, Europe, and Oceania as a dietary supplement owing to their high nutritional value [15, 16]. In the south and mid-west regions of Brazil, for example, the leaves of this plant, known locally as serralha, chicória-brava, and serralheira [17, 18], have a bitter taste resembling spinach and are used in salads [19]. Moreover, in several American countries, countless cultures have utilized *S*. *oleraceus* in a medicinal capacity to treat hepatitis, headaches, nephropathies, stomachaches, and ulcers [20, 21].

In Brazilian traditional medicine, the roots, leaves, and inflorescences of *S*. *oleraceus* are popularly used orally in the form of infusions or decoctions to treat stomachaches and other gastrointestinal disturbances [20, 22–24] and are also widely used as a depurative and laxative [25], an anti-inflammatory agent [26, 27], and in the treatment of cardiovascular problems. Indeed, some experimental studies have validated the popular use of *S*. *oleraceus* concerning its anxiolytic [18], anti-inflammatory [28, 29], and antitumor [30] properties.

Based on the widespread use of the leaves of *S*. *oleraceus* in the treatment of stomach diseases [22, 23], the present study was designed to be the first experimental investigation of the gastroprotective mode of action of this species. Specifically, we sought to validate the popular use of *S*. *oleraceus* as a natural anti-ulcerative resource and to evaluate the mode of action of a hydroalcoholic extract of the leaves of this plant.

## 2. Methods

### 2.1. Plant Material

The aerial parts of *S*. *oleraceus* were collected in Chapecó (SC), Brazil (27°01′55.14′S and 52° 47′29.42′′O), in September of 2018. The Professor Adriano Dias de Oliveira, curator of the Herbarium of the Community University of the Region of Chapecó (Unochapecó), verified the plant species and a voucher specimen was deposited (#3701).

### 2.2. Extract Production

The samples of *S*. *oleraceus* were dried at 25 ± 5°C and pounded in a knife mill (Ciemlab®, CE430), passed through a sieve (425 *μ*m), identified, and kept protected from light. To produce the extract hydroalcoholic (HES), dry-milled *S*. *oleraceus*'s leaves were macerated during five days with 70% ethanol 70% (0.02 w/v). The HES was filtered and concentrated using evaporation.

### 2.3. Evaluation of the Total Flavonoid Amount

The quantification of total flavonoids was measured by Woisky and Salatino [31], with adequations. In brief, 1 mL of the HES solubilized in methanol at a concentration of 1000 *μ*g/mL was added to 1 mL of AlCl_3_ 2% also solubilized in methanol and after 60 min the spectrophotometer readings were performed at 365 nm. To provide the calibration curve, quercetin was diluted in methanol as a standard (10, 15, 20, 25, and 30 *μ*g/mL), and the readings were also performed in triplicate. The quantification of flavonoids was described in mg/g of extract.

### 2.4. Mass Spectrometry Analysis (ESI-IT-MS^n^)

The direct injections of the HES were performed on the Thermo LTQ-XL apparatus (IT-MS) equipped with an electrospray ionization (ESI) source, in negative mode, with tubing at 280°C, spray voltage of 5.00 kV, capillary voltage of –35 V, and a tube lens of –100 V, with a flow sample of 10 *μ*L/min. The fragmentations within the multiple stays were allotted through the collision-induced dissociation (CID) method with helium and a collision energy of 30 eV.

### 2.5. In Vitro Assay of Radical Scavenging Activity

The antioxidant potential of HES was evaluated in keeping with Brand-Williams [32]. The HES, vitamin C, gallic acids, and quercetin (15–250 *μ*g/mL), or water (negative control group), were mixed with 2,2-diphenyl-1-picrylhydrazyl (DPPH) methanolic solution at 400 *μ*g/mL. Subsequently, the samples were incubated. Then, the absorbances were read at 517 nm in triplicates, and values were expressed as IC_50_.

### 2.6. Animals

Male mice Swiss, 3 months old (20–35 g) and male rats Wistar, 3 months old (180–200 g) from the Central Animal House of Unochapecó were kept in propylene cages under 25°C and a 12-hour light/dark cycle, with food and water freely. All experiments were conducted following ARRIVE guidelines and the ethical principles for animal experimentation of the National Council for Animal Experimentation. The experiments were approved by the Institutional Animal Ethics Commission of Unochapecó (020/17, December of 2017). The animals were fasted for 12 h before the experiments with water *ad libitum*. All the experiments were performed after approval by the Institutional Animal Ethics Committee of Unochapecó (approval number 020/17, December of 2017). All in vivo experiments were done in triplicate.

### 2.7. Dose Response Study

In traditional usage, an infusion of *S*. *oleraceus* is usually prepared with 6.0 g of dried leaves in 150 mL of water and ingested thrice each day by oral route, totaling an intake of 450 mL of infusion by day. Supporting this data, the first 450 mL of an infusion was prepared following this proportion in vegetal material and water, and its dry residue was calculated, reaching 2.3 g. Therefore, someone with 80 kg weight and using 450 mL of this infusion by day will receive approximately 29 mg/kg/day. Given this value, HES was tested at a dose of 30 mg/kg and at a dose 10 times greater and another 10 times less, i.e., 300 and 3 mg/kg, ensuring doses in a logarithmic scale as well as verifying the dose response.

### 2.8. Evaluation of Gastroprotective Activity

#### 2.8.1. Acidified Ethanol-Induced Gastric Ulceration

After 12 h of fasting, mice were divided into six groups (each containing six individuals) and orally pretreated, except the naïve group) with vehicle (Veh: saline plus 1% tween-80, 1 mL/kg), carbenoxolone (CBX: 200 mg/kg), or HES (3, 30, or 300 mg/kg) 1 h before the intake of acidified ethanol (0.3 M HCl in 60% ethanol, 0.1 mL/10 g). At 1 h after ulcerogenic administration, the mice were euthanized using thiopental (140 mg/kg, i.p.). The stomachs were removed to measure the ulcer area using EARPs software® [33]. This experiment was done in triplicate.

#### 2.8.2. Histological and Histochemical Evaluation

The ulcerated gastric tissue was removed and properly fixed for 24 h. To produce the slices, the tissues were dehydrated, embedded in paraffin, sectioned at 5 *μ*m, deparaffinized and some slides were stained with hematoxylin/eosin (HE). A score was employed to quantify histological alterations in the ulcerated mucosa. Briefly, 1 cm of every histological section was examined for epithelium loss (score: 0–3), edema within the upper mucosa (score: 0–4), hemorrhagic damage (score: 0–4), and also the presence of inflammatory cells (score: 0–3). The slices were analyzed by an independent pathologist in a blind manner. Further, the remaining histological slides were used for histochemical analysis of mucins using the periodic acid Schiff (PAS) method, which stains glycoproteins like mucins in pink, as earlier performed [34].

#### 2.8.3. Biochemical Analysis of Gastric Tissue

A homogenate was prepared with ulcerated tissues using 200 mM potassium phosphate buffer (pH 6.5) and the levels of reduced glutathione (GSH) was measured as previously described [35]. Another portion of the homogenate was centrifuged under 9000 × *g*, at 4°C by 20 min to get a supernatant, which was employed to see the activities of superoxide dismutase (SOD) [36], catalase (CAT) [37], and glutathione-*S*-transferase (GST) [38]. Besides, aliquots of the supernatant were employed to determine the content of tumor necrosis factor alpha (TNF) using ELISA kits (*R* & *D* Systems®, Minneapolis, MN) in accordance with the manufacturer's instructions. The precipitate was resuspended and centrifuged at 11000 × *g* for 20 min at 4°C to get a supernatant used to determine the activity of myeloperoxidase (MPO), as described by Young [39].

### 2.9. Determination of Gastric Secretion

Gastric secretion was assayed as described previously by Shay et al. [40]. The animals were treated intraduodenally with vehicle (Veh: 1 mL/kg, *n* = 6), HES (300 mg/kg, *n* = 6), or omeprazole (Ome: 20 mg/kg; administered orally 30 min before the ligature, *n* = 5). The animals were placed under 3% isoflurane anesthesia, during which the abdomen was opened for the procedure of pylorus ligation. At 4 h postligature, the animals were euthanized, the stomach was opened, and the gastric secretions were collected. Having measured the amount of volume employing a graduate tube, pH using a pH meter, and total acid content by titrating with NaOH (0.01 N) using phenolphthalein as an acid–basic indicator. The results were expressed as mL, pH, and Eq [H^+^]/mL, respectively. This experiment was done in triplicate.

#### 2.9.1. Estimation of Pepsin Activity

To estimate pepsin activity in gastric contents, we adopted the technique utilized by Silva [41]. Aliquots of digestive juice (100 *μ*L) from animals subjected to pyloric ligation were mixed with 500 *μ*L of acidified bovine albumin (5 mg/mL in 0.06 N HCl) and incubated at 37°C for 20 min, after which hydrolysis was terminated by the addition 500 *μ*L of 10% trichloroacetic acid. Then, the samples were centrifuged at 176 × *g* for 20 min, and 1 mL of the supernatant was added with 5 mL of 0.5 M sodium carbonate and 500 *μ*L of 1 N Folin-Ciocalteu reagent. Further, the absorbance was measured at 600 and results were calculated employing a standard tyrosine curve (30–1000 millimoles/mL) because pepsin cleaves albumin releasing tyrosine residues and expressed in terms of millimoles of tyrosine/mL.

### 2.10. Statistical Analysis

Statistically significant differences between groups were calculated using one-way analysis of variance (ANOVA) followed by the Bonferroni's post-test to parametric data. Nonparametric data were expressed as median with interquartile range and analyzed by Kruskal–Wallis followed by Dunn's test. The software GraphPad version 8.00 for Windows (GraphPad Software, La Jolla, CA, USA) was used. The values were represented by means ± standard error of the means (S.E.M) and *p*values less than 0.05 (*p* < 0.05) were considered significative.

## 3. Results

### 3.1. Chemical Analysis

#### 3.1.1. Quantification of Flavonoids

Analysis though of spectrometric UV/Vis using calibration curve the quercetin (10–30 *μ*g/mL; *y* = 0.0614*x* − 0.0384; *R*^2^ = 0.9973) showed high amount flavonoids in the hydroalcoholic extract of *S*. *oleraceus* (67.0 mg/g; 6.7%).

#### 3.1.2. Mass Spectrometry Analysis

The hydroalcoholic extract of *S*. *oleraceus* (HES) obtained in the present study was analyzed by tandem mass spectrometry using an electrospray ionization source coupled to an ion trap mass spectrometer analyzer based on a direct infusion technique. The structures of the constituent compounds were determined based on their MS_2_ and MS_3_ fragmentation patterns and compared with literature data. The presence of the flavonoid luteolin-7-*O*-*β*-D-glucoside, a characteristic compound of the species, was annotated, giving the [*M*-*H*]^−^ ion at *m/z* 447. The MS_2_ fragmentation of the precursor ion at *m/z* 447 led to a product ion at *m/z* 285 [*M*-162-*H*]^−^ (loss of glucose). The MS_3_ fragmentation of the parent ion at *m/z* 285 gives the products ions at *m/z* 285, 226, 257, 217, 241 and 198 [42, 43].  Table 1 and Figure 1 summarizes the results of the annotation of compounds by mass spectrometry, finding the fragmentation patterns of other glycosylated phenolic compounds, such as caffeoyl glucoside, quercetin glucoside, and kaempferol glucoside, as well as the aglycones of luteolin, kaempferol, quinic acid, ellagic acid, and rhamnetin [43–45].

#### 3.1.3. In Vitro Scavenging Activity of HES

The antioxidant activities of HES (15–250 *μ*g/mL) and the positive controls (gallic acid, ascorbic acid, and quercetin) were determined based on the DPPH scavenger assay. HES was found to have a half-maximal inhibitory concentration (IC_50_) of 15.41 *μ*g/mL, confirming its antioxidant capacity *in vitro*. In line with expectations, gallic and ascorbic acids and quercetin also showed significant effects in reducing DPPH, with IC_50_ values of 3.27, 8.9, and 12.2 *μ*g/mL, respectively.

### 3.2. Effects of HES on Acidified Ethanol-Induced Gastric Ulceration

Whereas the acidified ethanol-ulcerated mice treated with vehicle showed severe damage to the gastric mucosa, those receiving HES (3, 30, or 300 mg/kg) showed reductions in the size of the ulcerated area by 39, 71.5, and 76.2%, respectively, compared with the vehicle-treated mice (*p* < 0.05, *p* < 0.001, and *p* < 0.001, respectively), which was found to be comparable to the reduction in size observed in mice treated with positive control CBX (Figure 2(a)). Representative macroscopic images of the ulcerated tissues from animals in each group are presented in Figure 2(b).

Observation of histological preparations revealed that ulcerated mice presented intense damage with epithelial loss and hemorrhagic lesions reaching a score value with median equal to 9.0; whereas mice treated with HES at 30 (*p* < 0.01) or 300 mg/kg (*p* < 0.001) or CBX (*p* < 0.05) were characterized by fewer structural disruption to the gastric mucosa, compared with vehicle-ulcerated mice (Figure 3(a)). Images of the tissues obtained from mice in all experimental groups, which were subjected to histological staining with hematoxylin and eosin, are shown in Figure 3(b).

Furthermore, compared with vehicle-ulcerated mice, we also detected an elevation in the PAS-staining to glycoproteins like mucins of mice treated with HES at doses of 30 and 300 mg/kg by 361.4 and 477.5%, when compared to vehicle-ulcerated group (*p* < 0.001) (Figure 4(a)). Representative images of PAS-staining are depicted in Figure 4(b).

### 3.3. Effect of HES in the Levels of GSH and TNF and Activities of GST, SOD, CAT, and MPO

As shown in Table 2, the administration of acidified ethanol reduced SOD activity and GSH levels, which was prevented in mice treated with HES (300 mg/kg) compared with the vehicle-ulcerated group (*p* < 0.01). Moreover, the observed effect was found to be superior to that obtained in mice treated with carbenoxolone (*p* < 0.05). Similarly, compared with the vehicle-ulcerated group, HES (300 mg/kg) treatment had the effect of increasing the activities of GST and CAT (*p* < 0.01), whereas MPO activity, evaluated as an indication of neutrophil migration, was reduced by treatment with both HES (300 mg/kg) and carbenoxolone (*p* < 0.01). The effects of HES (300 mg/kg) on inflammatory markers were further reinforced by a 43% reduction in the TNF levels compared with those in the vehicle-ulcerated group (*p* < 0.01) (Table 2).

### 3.4. Effect of HES in the Gastric Acid Secretion Parameters of Rats

Our analysis of the gastric acid secretion in pylorus-ligated rats revealed that, on average, those in the vehicle-treated group secreted 7.54 ± 0.65 mL of gastric juice, the pH of which was equal to 1.92 ± 0.26, reaching a total acidity of 0.036 ± 0.006 Eq [H^+^]/mL, and with a peptic activity of 4.74 ± 0.81 *μ*M of tyrosine/mL. Interestingly, although no significant change in the volume of secreted gastric acid was observed in rats administered HES (300 mg/kg, i.d.), we detected an increase in pH and a corresponding reduction in gastric acidity and the activity of pepsin compared to the vehicle group (*p* < 0.05). Similarly, in accordance with expectations, we observed an increase in the pH and reductions in the acidity and peptic activity of gastric acid secretions in rats treated with the proton pump inhibitor omeprazole at a dose of 20 mg/kg (*p* < 0.05) (Table 3).

## 4. Discussion

*S*. *oleraceus* is consumed worldwide for its nutritional properties and efficacy in the treatment of digestive diseases and other ailments [16, 18, 23, 46]. Although there are preliminary reports on the anti-ulcerogenic effects of extracts and fractions of *S*. *oleraceus* [47], the gastroprotective mode of action of polar extracts (which are more comparable to the preparations consumed in popular usage) of the leaves of this medicinal plant has yet to be sufficiently investigated. Accordingly, we believe that the present study is the first to demonstrate the significant gastroprotective effects of pretreatment with HES in mice with acidified ethanol-induced gastric ulceration. Moreover, we show that this reduction in gastric damage involves an increase in antioxidant defense mechanisms, both enzymatic and non-enzymatic, as well as the reduction in neutrophil migration or pro-inflammatory cytokine TNF secretion. In addition, HES pretreatment was found to be associated with an increase in the pH of gastric acid secretions and, in turn, reduced gastric acidity and peptic activity. Moreover, we suspect that these effects may, in part at least, be attributable to the activity of certain polyphenolic compounds as the flavonoids, including luteolin-7-*O*-*β*-D-glucoside, identified in HES.

Ethanol has been established to play a key role in gastric mucosal ulcerations, given that it induces gastric ulceration via several mechanisms, including depletion in the levels of gastric mucus and bicarbonate, and damage to phospholipid layers caused by an exacerbated generation of ROS and the subsequent intense inflammatory response [6]. In line with expectations, we found that macroscopically, vehicle-treated mice bearing acidified ethanol-induced ulcers had a larger extent of a lesioned area characterized by hemorrhagic stripes, which microscopically was evidenced by an extensive breakdown of the gastric epithelium. However, the pretreatment with HES was associated with a significant reduction in the size of the lesioned area, comparable to the results obtained with carbenoxolone, which was used as a positive control. Moreover, histological analysis confirmed that HES was effective in maintaining the integrity of the gastric mucosa, notably in those mice treated with 300 mg/kg HES, thereby preventing hemorrhagic injury and epithelial cell loss [48, 49].

Previous studies have demonstrated that the alcoholic extracts (95% ethanol) obtained by percolation and *n*-butanol fractions from the roots and aerial parts of *S*. *oleraceus* showed antiulcerogenic activity (250 and 500 mg/kg) [47]. However, the tests realized were very preliminary and so far, the gastroprotective mode of action is not known. Considering that understanding how the diverse chemical components in medicinal herbs contribute to the overall pharmacological effect is a major challenge for current studies, and that offers new possibilities for investigating the explicit targets [50], this work advanced the comprehension of the gastroprotective pharmacological mechanism for preparations that mimic popular use with leaves of the plant.

In addition, extracts of *S*. *oleraceus* have anti-inflammatory and anti-edematogenic effects, and these effects are mainly associated with certain phenolic compounds in this plant, which have a cytoprotective activity that can ameliorate the inflammatory response [28, 51]. The gastroprotective activity of HES and the anti-inflammatory properties of *S*. *oleraceus* extracts accordingly mark this medicinal species as a beneficial pharmacological alternative to the currently available anti-inflammatory resources.

Based on augmented periodic acid-Schiff staining, we also detected an increase in the glycoprotein content of the gastric mucosa in mice treated with 30 and 300 mg/kg HES. Concerning gastric injuries, the secretion of mucus represents an essential protective factor, in that it contributes to preventing the direct contact between these cells and digestive enzymes and other potentially harmful agents [51]. Indeed, although probably not the only pharmacological mechanism underlying the gastroprotective activity of HES, there is evidence that mucus secretion is one of the main events associated with these effects.

It is well established that ethanol-induced ulceration promotes an increase in ROS production and, in turn, gives rise to oxidative stress and cell death [52]. In this regard, reduced glutathione (GSH) is a component of the first line of antioxidant defense that is used as a marker of the antioxidant capacity of biological systems. In the present study, we observed an evident depletion of GSH levels in vehicle-treated ulcerated mice in response to the oxidative insult promoted by ethanol, which, interestingly, was prevented by pretreatment with 300 mg/kg HES. Corroborating these findings, previous studies have reported the protective effect of preparations from *Sonchus asper* L. against GSH depletion associated with potassium bromate-induced reproductive stress in male rats [53], CCl_4_-induced hepatotoxicity [54], and in the brains of rats [55]. Furthermore, since our DPPH assay results, it can be inferred that the scavenging activity of HES constituents can contribute to the neutralization of ROS and preservation of GSH reserves, which is consistent with the findings of Yin [15], who demonstrated the nitrite, hydroxyl, and DPPH radical scavenging activities of hydroalcoholic extracts of *S*. *oleraceus*.

GSH also serves as a cofactor for GST enzymes, which are dimeric proteins that play multiple biological roles [55]. Thus, the observed increase in GST activity in response to treatment with 300 mg/kg HES could be seen as indicative of enhanced bioavailability of GSH in this group, thereby reflecting an augmentation of gastric mucosa protection against cytotoxic agents.

Among the multiple types of ROS generated in mammals, superoxide anions, hydrogen peroxide, and hydroxyl radicals are the principal types targeting the gastric mucosa. As countermeasures, however, the body has a suite of enzymatic antioxidants with which it mounts a defense against this insult. Superoxide anion, for example, is dismutated by superoxide dismutases (SODs), yielding oxygen and hydrogen peroxide [56], whereas CAT subsequently promotes the conversion of hydrogen peroxide to water and oxygen [57]. Like the observations of Costa [55], although we found that SOD activity remained essentially unaltered in the vehicle-treated ulcerated mice, there was a detectable reduction in the activities of CAT and GST, as evidenced by an attenuation of the mucosal defenses against peroxides and xenobiotics. In agreement with other studies [58], we found that ethanol intake reduces SOD activity. Moreover, the administration of 300 mg/kg HES increased the activities of SOD and CAT to levels higher than the basal levels found in non-ulcerated animals. Despite its gastroprotective properties, the administration of CBX did not increase the SOD. Furthermore, Teugwa [1] has reported that whole-plant hydroethanolic extracts of *S*. *oleraceus* have a beneficial effect on diabetic rats, associated with a substantial increase in CAT activity in the kidney and liver of these animals. Collectively, our analyses of the antioxidant properties of HES, both *in vitro* and in a biologically complex system, provide compelling evidence that this natural preparation can serve as a beneficial agent with marked antioxidant activity, thereby justifying its widespread use in traditional medicine practiced worldwide.

Inflammatory processes, including the ulcer induced by ethanol, are characterized by elevated levels of neutrophils and inflammatory cytokines [59], and in this regard, given that MPO is stored within neutrophil granules, the determination of this enzyme's activity has been employed as an indirect indicator of neutrophil accumulation in ulcerated tissues [60, 61]. In the present study, we found that the administration of HES resulted in a reduction in MPO activity, thereby indicating the inhibition of neutrophil infiltration into the mucosa and, consequently, a reduction in gastric tissue inflammation. The beneficial effects of HES concerning inflammatory markers were confirmed through our analysis of TNF levels in ulcerated mice. TNF plays an important role in the generalized inflammatory process by activating neutrophils [62], and we found that 300 mg/kg HES was effective in reducing TNF accumulation in ulcerated tissues. These observations are consistent with those reported by Vilela [20], who found that a hydroethanolic extract of *S*. *oleraceus* inhibited leukocyte recruitment into the peritoneal cavity of rats exposed to carrageenan.

Given the importance of gastric acid secretion in ulcer pathogenesis and therapy, we examined the effect of HES on basal secretion in pylorus-ligated rats. Interestingly, we found that whereas at a dose of 300 mg/kg, HES did not reduce the volume of gastric acid secreted, comparable with the effects of the positive control omeprazole, it did have the effect of increasing secretion pH and thereby resulted in reductions in lumen content, gastric acidity, and peptic activity. However, the mechanisms underlying the antisecretory properties of HES require further investigation.

The pharmacological effects attributable to HES appear to be associated with the activity of polyphenols and flavonoids such as luteolin-7-*O*-*β*-D-glucoside, annotated in our chemical analyses of the extract. It has widely been established that a diverse range of flavonoids have *in vivo* antiulcerative activity [63]. Furthermore, these compounds have been found to have marked antisecretory activity in pylorus-ligated rats, and it has been established that the primary mechanism of the anti-ulcerative activity of flavonoids can be attributed to their antioxidant properties, including the elimination of free radicals, chelation of metal ions, promotion of the activities of enzymatic and non-enzymatic antioxidants, and a reduction in lipid peroxidation. These activities appear to be associated with the presence of catechol rings, notably the double bonds between positions 2 and 3, and hydroxyl groups at positions 3, 5, and 7 [64]. Likewise, the polyphenols pointed out in this study (quinic acid, ellagic acid, and caffeoyl glucoside) are known to activate the endogenous antioxidant system and thus effectively scavenge excessive free radicals. Furthermore, these molecules can act as natural metal chelators and suppress free radical generation and lipid peroxidation in humans [65]. In addition, polyphenols demonstrate several biological functions, which include anti-inflammatory, immunomodulatory, and gastroprotective properties [66].

## 5. Conclusion

The hydroalcoholic extract of *S*. *oleraceus* leaves has gastroprotective effects mediated via an enhancement of antioxidant defenses and mucilaginous barriers, in parallel with a reduction in the inflammatory process. These effects are conceivably achieved, at least in part, by a reduction in the acidity of gastric secretions associated with the activity of flavonoids such as the luteolin-7-*O*-*β*-D-glucoside content of HES. We therefore believe that the findings of this study make an important contribution and advance our current understanding of the underlying pharmacological mechanisms. In addition, this study contributes to the popular use of plants and to the prospection of new gastroprotective agents.

## Figures and Tables

**Figure 1:** Structures of compounds annotated by ESI-IT-MS^*n*^ in the hydroalcoholic extract from aerial parts of *Sonchus oleraceus* (HES).

**Figure 2:** Effect of the hydroalcoholic extract from *Sonchus oleraceus* (HES, 3–300 mg/kg) and carbenoxolone (CBX; 200 mg/kg) on the acidified ethanol-induced ulcer (mean ± SEM; *n* = 6). (a) Mice induced with acidified ethanol and treated with saline (Veh). One-way ANOVA followed by Bonferroni test. ^*∗*^*p* < 0.05 and ^*∗∗∗*^*p* < 0.001 compared to vehicle ulcerated (Veh) group. Representatives images from each group are shown in Panel (b).

**Figure 3:** Histological appearance of the gastric sections of the hydroalcoholic extract from *Sonchus oleraceus* (HES, 3–300 mg/kg) and carbenoxolone (CBX; 200 mg/kg) on the acidified ethanol-induced ulcer after hematoxylin/eosin staining (HE), and after Periodic acid-schiff (PAS)-stained mucin-like glycoproteins.

**Figure 4:** Quantification of PAS-stained mucin-like glycoproteins for the hydroalcoholic extract from *Sonchus oleraceus* (HES, 3–300 mg/kg) and carbenoxolone (CBX; 200 mg/kg) on the acidified ethanol-induced ulcer (mean ± S.E.M; *n* = 6). One-way ANOVA followed by Bonferroni test. ^*∗∗∗*^*p* < 0.001 compared with vehicle ulcerated (Veh) group.

**Table 1:** Phytochemical analysis of hydroalcoholic extract from aerial parts of *Sonchus oleraceus* (HES) by ESI-IT-MS/MSn^*a*^.

Compounds	*m/z* [*M*-*H*]^−^	MS_2_	MS_3_⟶MS^*n*^	Reference
Luteolin-7-*O*-*β*-D-glucoside	447	285	285, 226, 257, 217, 241, 198	[43]
Quinic acid	191	111, 173, 85, 127	—	[44]
Kaempferol	285	211, 127, 257, 151, 241	—	[44]
Luteolin	285	285, 226, 257, 217, 241, 198	—	[43]
Ellagic acid	301	257, 272, 283	—	[44]
Rhamnetin	315	300, 271, 193, 165, 121	—	[45]
Caffeoyl glucoside	377^*b*^	341	179, 161, 143, 149, 131	[43]
Quercetin glucoside	463	301	151, 179	[44]
Kaempferol diglucoside	609	285	447, 267, 241	[43]

^*a*^Spectra recorded in negative mode, ^*b*^[*M* + Cl-*H*]^−^.

**Table 2:** Effects of hydroalcoholic extract from *S*. *oleraceus* (HES) on oxidative and inflammatory parameters of ulcerated tissue.

	MPO	TNF	GSH	SOD	CAT	GST
Naïve	0.033 ± 0.006	124.4 ± 15.5	915.2 ± 238.4	150.2 ± 13.6	17.57 ± 5.81	359.0 ± 13.1
Vehicle	0.097 ± 0.010^a^	589.9 ± 128.6^a^	1013 ± 116.2	109.8 ± 45.7^a^	6.73 ± 3.91	157.8 ± 17.4
CBX	0.041 ± 0.004^b^	293.5 ± 41.65^b^	1829 ± 96.1^ab^	106.3 ± 7.8	55.03 ± 5.91^ab^	325.1 ± 35.4^b^
HES	0.050 ± 0.006^b^	229.5 ± 20.15^b^	2547 ± 127.9^abc^	157.6 ± 13.8^abc^	41.39 ± 5.76^ab^	410.3 ± 46.3^b^

*Note.* Carbonoxolone (CBX, 200 mg/kg); hydroalcoholic extract of *S*. *oleraceus* (HES, 300 mg/kg); myeloperoxidase (MPO, mD.O/mg of protein); reduced glutathione (GSH, *μ*g/mg of tissue); superoxide dismutase (SOD, U/mg of protein); catalase (CAT, *μ*mol/min/mg of protein), tumor necrosis factor (TNF), and glutathione S-transferase (GST, *μ*mol/min/mg of protein). Values are expressed as means ± S.E.M (*n* = 6). One-way ANOVA followed by Bonferroni's test. ^*a*^*p* < 0.05 vs. naïve group. ^*b*^*p* < 0.01 vs vehicle-treated group. ^*c*^*p* < 0.01 vs carbenoxolone group.

**Table 3:** Effects of HES on gastric acid secretion.

				
Vehicle	7.54 ± 0.65	0.0360 ± 0.0066	1.92 ± 0.26	6.47 ± 0.70
Omeprazole	6.62 ± 0.80	0.0092 ± 0.0040^*a*^	5.84 ± 1.11^*a*^	4.08 ± 0.18^*a*^
HES	7.58 ± 0.89	0.0137 ± 0.0045^*a*^	5.53 ± 0.99^*a*^	2.35 ± 0.57^*b*^

*Note.* Vehicle (0, 1 mg/kg), omeprazole (20 mg/kg), HES (300 mg/kg); volume (mL); total acidity (Eq [*H*^+^]/mL); peptic activity (mmol of tyrosine/mL). Values are expressed as means ± S.E.M (*n* = 5–6). One-way ANOVA followed by Bonferroni's test. ^*a*^*p* < 0.05 and ^*b*^*p* < 0.001 vs vehicle-treated group.

## Data Availability

The articles, images, and analysis tables used to support the findings of this study are available from the corresponding author upon request.
